The article "A Survey of Museum Applied Research Based on Mobile Augmented Reality" was published in 2022. Journal: Comput Intell Neurosci.

# A Survey of Museum Applied Research Based on Mobile Augmented Reality

**DOI:** 10.1155/2022/2926241

**Published:** 2022-08-17

**Authors:** Chong Wang, Ye Zhu

**Affiliations:** ^1^School of Art and Design, Guilin University of Electronic Technology, Guilin 450305, China; ^2^School of Business, Guilin University of Electronic Technology, Guilin 450305, China

## Abstract

Museums are the important places of education for preservation and dissemination of human material and intangible heritage. Nowadays, there are many problems in museums such as single display mode and fixed interaction style of collections, which makes cognitive load higher and visiting experience poorer for tourists. Mobile Augmented Reality is a technology that seamlessly integrates virtual information with real environment based on mobile devices. Museum applications based on Mobile Augmented Reality can improve the display richness and meet new visiting needs of the public in the digital era. Firstly, this article introduces the key technologies of Mobile Augmented Reality and its use in museums. Secondly, according to different application functions, classifiable explanations for Mobile Augmented Reality application examples are given. Thirdly, based on the progress in the application of Mobile Augmented Reality in museums at home and abroad, from three dimensions of content, guide, and interaction, designing thought regarding the application of Mobile Augmented Reality for museums is summarized.

## 1. Introduction

Museums are the important places for preservation, dissemination, and exhibition of human cultural heritage, and they aim at providing historical, cultural, and educational knowledge of various cultural relics for the public [1]. At present, collections in museums are mainly displayed in showcases with literal statement and the limited space in museums could not meet the needs of display of diversified cultural relics; the mode of interaction with the visitors is relatively single, and the behavior pattern tends to be fixed, without freshness and sensory stimulation, which may lead to higher cognitive load and reduced attention, thus causing poor visiting experience in museums. As shown in the data released by the National Cultural Heritage Administration, in 2019, the annual reception of 83% of the museums was 300,000 person-times or less; large museums were “bustling with visitors,” while the vast majority of small and medium-sized museums were “stagnant”; therefore, the degree of many small and medium-sized museums display could not meet the growing cultural needs of users. Under the background that museums are rich in resources, but their displays cannot meet the cultural needs of the public, digital transformation of museums should be performed, for new technologies can endow multidimensional display space for the exhibits, meet the deeper tourism needs of users in the new era, and help to promote and inherit the culture.

The article "A Survey of Museum Applied Research Based on Mobile Augmented Reality" was published in 2022. Journal: Comput Intell Neurosci.

Augmented Reality is a technology that seamlessly integrates virtual information with real environment based on a device screen or an entity mapping, which can improve people's experience, feeling, and cognition of the real world [2]. Based on display modes, Augmented Reality can be divided into head-mounted display, handheld display, and space display [3], while Mobile Augmented Reality (MAR) is a technology that adopts the mode of display with handheld smart devices or head-mounted display [4], which, with great potential in industries such as cultural travel, entertainment, manufacturing, and education, is high in business value and practical value.

Museum application based on Mobile Augmented Reality can make collection information digitized and integrate virtual information of cultural relics such as texts, animations, models, and audio in the real context [5]; therefore, it can stimulate the senses of the users in a more natural and vivid way and make up for the information faulty. As a result, visitors can get richer knowledge and more novel experience and can also achieve real-time interactive participation. Augmented Reality applied in museums can fully express the cultural deposits and humanistic connotation of the collections and also improve the experience quality and educational effect from the perspective of the individual users.

This article firstly introduces three key technologies of the MAR system (tracking registration, real-time interaction, and virtual-real fusion) and summarizes their application in the field of museums. Secondly, the application examples of MAR from the aspects of sensory stimulation, behavioral pattern, and interactive experience are described. Finally, this paper summarizes the design ideas of MAR application from the dimensions of content design, guide design, and the interaction design based on research cases.

## 2. Key Technologies of Mobile Augmented Reality and Their Application in Museums

In 1992, Caudell et al. [6] first proposed the term “Augmented Reality” in a maintenance project of Boeing aircraft, and then the concept of AR started attracting people's attention. Milgram and Kishino [7] originally expressed the relationship between real world, Augmented Reality, and Virtual Reality in a taxonomic manner; Augmented Reality refers to a state of incomplete immersion between physical environment and virtual fantasy. While receiving virtual information which is diversified and dynamic, the users can maintain the perception of reality. ARToolKit, the first Open Source architecture of Augmented Reality, was created in 1999 and opened the door for software developers to use Augmented Reality. Azuma pointed out the technical characteristics of the Augmented Reality system such as tracking registration, real-time interaction, and virtual-real fusion [2]. The MAR system can achieve registration of virtual objects by real-time tracking of the surrounding environment, present virtual-real fusion with display devices, and achieve interaction with virtual objects using the real-time interaction technology. The overall architecture is shown in Figure 1.

The article "A Survey of Museum Applied Research Based on Mobile Augmented Reality" was published in 2022. Journal: Comput Intell Neurosci.

### 2.1. Tracking Registration Technology and its Application

Tracking registration refers to the technology that can realize the mapping of virtual and real space coordinate system by tracking the viewpoint and field of view of a user and superimpose virtual information in the real scenario according to the accurate spatial perspective relationship [8]. At present, there are three types of tracking registration techniques: vision-based tracking registration technology, hardware sensor-based tracking registration technology, and hybrid tracking registration technology. The classification is shown in Figure 2.

#### 2.1.1. Vision-Based Tracking Registration Methods

The tracking registration methods based on computer vision mainly complete tracking registration of virtual information through processing the images captured by a camera window; they are mainly divided into the marker-based and natural feature-based methods [8].

*(1) Marker-Based Tracking Registration Method*. When using the tag-based approach, we should place the tags with internal code in the environment in advance, which can make users scan the image datum and coding feature of the markers, so as to complete the transformation of the coordinate system between virtual space and real space according to the affine invariance principle [9]. This method has strong stability, but there may be problems such as failure in identification and object drift when any marker is blocked. For example, through scanning the identification code on the book “Exploitation of the Works of Nature,” the user may view 3D models of ancient utensils in China. Through scanning the black and white markers in the American Museum of Natural History, user may watch the short film regarding the space exploration. And through scanning the marker next to the artifact in the Celtic Heritage Museum, there would be a “virtual Celt” who can talk about historical stories [10] (Figure 3).

*(2) Natural Feature-Based Tracking Registration Method*. Natural feature-based tracking registration method (without any marker) can identify natural feature points in the environment with the feature extraction algorithm, to realize camera pose mapping. This method requires neither a marked object nor cognitive transcendence of the user. Natural feature-based tracking registration method involves edge detection, point of interest tracking, template matching, optical flow tracking, depth imaging, and Model-free tracking (Table 1) [11], and the commonly used algorithms include SIFT, SURF, FAST, ORB, and BRIEF.

The article "A Survey of Museum Applied Research Based on Mobile Augmented Reality" was published in 2022. Journal: Comput Intell Neurosci.

Natural feature-based method is susceptible to the changes in the exhibit location, light intensity, and reflectivity. Purnomo et al. [18] discussed the impact of distance, angle, and light intensity in cloud recognition of 3D feature points on recognition effect based on Sangiran Museum. The results indicated that the greater scanning angle would reduce the recognition distance, and the greater distance of light intensity would widen the range of recognition; the average maximum tilt angle for keeping the object stable was determined as 25 degrees. Khan et al. [19] identified and tracked the exhibits with the Deep Learning Algorithm. Firstly, they identified the images and constructed a data set of cultural relics with the Convolutional Neural Network and back propagation algorithm. Secondly, they captured the data of the camera frame to obtain the tags of cultural relics, thus retrieving the corresponding information in the database. Sugiura et al. [20] evaluated the usability of the identification methods with and without markers based on the Museum of Medical Specimens (Figure 4), and the results indicated that the marker-based method would influence the appearance of the exhibits and interfere with the behavior of visiting, while the natural feature-based method may be stronger in usability.

#### 2.1.2. Hybrid Tracking Registration Method Based on Vision and Hardware

The hardware-based tracking registration method can obtain user space location transfer data to adjust the pose and complete the registration based on the technologies such as acoustic tracking, optical tracking, magnetic sensor tracking, and inertial sensor tracking. This method is highly real-time, but there are multiple factors affecting the effect of sensors, and they may result in relatively low precision of tracking registration; for example, when the time of arrival (ToA) of sound is used for acoustic tracking, the speed of sound will affect the tracking precision due to the temperature and humidity; magnetic sensor tracking would shake due to the increased sensing distance and electromagnetic noise, thus leading to a certain loss of certain precision [11]. Vision-based tracking registration method has high precision, but greater system delay. The hybrid tracking registration technology can combine the two technologies and complement each other's advantages; with the hardware for real-time tracking to obtain spatial information, and visual algorithm for 3D calibration, this method can ensure high system robustness and registration precision. For example, the hybrid tracking method can prevent the failure in visual tracking under cover and solve the problem of difficult edge detection and tracking due to partial loss of cultural relics and outdoor light changes [11].

The article "A Survey of Museum Applied Research Based on Mobile Augmented Reality" was published in 2022. Journal: Comput Intell Neurosci.

Miyashita et al. [21], based on marker-free tracking and rotation sensor, prepared MAR demonstration for Islamic Art Exhibition, but the tracking area of the system was limited to the periphery of six points, which restricted the range of user experience. Hammady et al. [22] combined the SLAM marker-free tracking method with indoor positioning beacon and established communication among the devices and the server based on IBeacons low-power Bluetooth communication function. Tsai et al. [23] designed MAR navigation with the image recognition and beacon sensing technology (Figure 5) and set multiple guides based on beacon positioning, to meet the needs of users for exhibit explanation and floor navigation. Sun et al. [24] designed a method of intelligent spacing selection model, which can improve the problems of high delay and high energy consumption in the Internet of Things. This method can better prevent interference in the process of information transmission in the museum Internet of Things.

### 2.2. Real-Time Interaction Technology and Its Application

MAR real-time interaction mainly involves the interaction with a 2D screen and control of 3D virtual objects. The scholars mainly focused on the control of 3D objects. MAR system mainly involves the following interactions: touch-based interaction, air gesture-based interaction, and device-based interaction.

#### 2.2.1. Touch-Based Interaction

Touch-based interaction controls 3D objects by processing the position data of fingertips on the screen. Due to the limitation of movement of fingers, small screens of mobile devices, and limited touch range, most MAR applications remove the functions of translational motion and zooming but maintain rotation only, or separate translational motion and rotation by mode switching. Vogel and Baudisch [25] first proposed the use of shifting to get rid of the problem of object covering by fingers on small touch screens; he displayed the contents covered by fingers near the position of touching. Abbas et al. [26] proposed a calculation method converting 2D screen coordinates to 3D virtual coordinates, but this system may result in errors due to the failure in accurately picking up the center pixel on a small screen. In addition, the user needs to support the device with one hand to keep tracking and realize virtual interaction with the other hand; this touch behavior would cause certain movement of the camera, leading to a negative impact on tracking precision and user experience. Bai et al. [27] designed the mode of freeze view (Figure 6); in this mode, the system would lock the current camera frame, stop the visual tracking of reality, and save the current resources. The user can operate freely, without affecting the tracking effect by shaking upon touching; however, the static view would reduce the sense of real-time engagement.

The article "A Survey of Museum Applied Research Based on Mobile Augmented Reality" was published in 2022. Journal: Comput Intell Neurosci.

#### 2.2.2. Gesture-Based Interaction

Gesture-based interaction is a mode of selecting and controlling virtual objects through tracking and recognizing natural gestures. Its core techniques mainly include gesture segmentation, gesture analysis, and gesture recognition. Seo et al. [28] took palm as a marker and controlled 3D objects by moving and rotating the palm. Chun and Hollerer [29] used texture mapping and background subtraction to accurately detect finger gestures and avoid self-covering. Bai et al. [27] identified the projection points and polygons of fingertip mapping by a RGB depth camera and marked and tracked the prominent fingertips. As for MAR application in museums, there are various problems of covering during gesture-based interaction, and the covered contents should be identified by a lot of auxiliary depth data; meanwhile, due to the limited motion range of hands, long-term interaction would lead to user fatigue.

#### 2.2.3. Device-Based Interaction

Device-based interaction is a mode using built-in sensors to map the positions of 3D objects; the user may move or rotate the 3D objects with a handheld mobile device. Although there is high robustness, the user should watch the screen in a real-time manner and should not perform large-scale rotation of the device. Samini and Palmerius [30] designed two states of pressing and releasing, which can realize large-scale rotation through locking 3D objects; however, frequent and excessive rotation would also lead to failure in tracking registration.

### 2.3. Virtual-Real Fusion Technology and Its Application

Virtual-real fusion refers to the display technology that seamlessly integrates virtual scenes with real ones. An Augmented Reality system should ensure the consistency of virtual and real scenes, including geometric consistency, illumination consistency, and time consistency. With Augmented Reality, characterized by virtual-real combination, the experiencers can be brought into a fictional space by virtual information such as images, models, and animations, which can create multilevel immersion for users, thus meeting their cultural needs for immersive experience.

The article "A Survey of Museum Applied Research Based on Mobile Augmented Reality" was published in 2022. Journal: Comput Intell Neurosci.

As shown in previous studies, Ultra-Mobile-PC, with certain computing and image processing capabilities, could be taken as then display device for MAR applications. Later, with the development of smart devices, handheld smart devices such as mobile phones and tablets, as well as head-mounted displays such as HoloLens and Google Glasses, have been the mainstream MAR application devices. Handheld smart devices could collect data from the real environment by camera, and the built-in information processing unit could recognize and processes the image, and perform tracking registration of real objects with a variety of embedded sensors (such as accelerometer, gyroscope, infrared sensor, and magnetometer), to integrate virtual images and real ones. Head-mounted displays are divided into video perspective and optical perspective displays, in which, video perspective displays have the similar principle of realization to handheld smart devices, while optical perspective displays can realize virtual-real fusion by the optical fusing device in front of the user. The optical fusion device can present partially transparent and partially reflected images. The transparent part allows users to see the real world, and the virtual image generated by the system can be projected into the user's eyes at the same time, so the user can see the combined virtual and real image.

The above two types of devices have their own advantages and disadvantages. The head-mounted display, due to the closeness to human eyes, can bring full immersion experience and get rid of manpower for holding a handheld device, but without a touch screen, there would be priori cost in the case of gesture interaction; at the same time, partial transmittance may reduce the display brightness and image quality. Handheld devices are small, light, and easy to carry, and the users may achieve interaction with touch screens; however, the users should hold the devices to target at the objects during visiting. Long-term holding would make the users tired. In terms of market potential, head-mounted displays have not reached the level of consumption due to the high cost, while handheld smart devices, with certain image processing ability and stable network collaboration ability, have a huge user base; therefore, they are the most potential MAR application devices at present.

### 2.4. Introduction of MAR Application SDK

At the 2019 AWE Augmented Reality Expo, MAR development tools were ranked according to the market support rate (Table 2). The ARKit framework of Apple Inc based on IOS system has many significant advantages and functional features and has the maximum support rate; the ARCore framework developed by Google Company supports Android devices, has a higher device base, and also has a higher support rate; Unity and Unreal have integrated the core functions of ARKit and ARCore SDK development packages as professional real-time content development platforms and further improved the efficiency of AR project development. Unity is committed to building a unified and open AR development platform with a higher support rate; Vuforia has always been an AR SDK favored by developers, with rich functions and stable and efficient identification technology. The study work of many scholars is based on AR Application developed by Vuforia; Spark AR of Facebook and Lens Studio of Snap are AR filters that favor social sharing; Sumerian of Amazon is a browser-based tool for building interactive 3D scenes, supporting all WebGL or WebVR graphics rendering browsers; based on the powerful digital content software ecosystem of Adobe, the Project Aero can quickly access the digital resources of Photoshop, Illustrator, Dimension, etc. to help developers build simple AR scenes and interactive experiences for ARKit. Furthermore, there are excellent AR SDK development packages, such as Sensetime Sense AR, Baidu's Du Mix AR, and Hi AR.

The article "A Survey of Museum Applied Research Based on Mobile Augmented Reality" was published in 2022. Journal: Comput Intell Neurosci.

## 3. Application Cases of Mobile Augmented Reality in Museums

In museums, there may be tangible cultural relics such as paintings, calligraphy, and architecture and intangible assets such as historical stories, folklores, and cultural customs. While focusing on the types of collections and visiting behaviors of users in museums, MAR applications can be divided into three categories: (1) The applications naturally integrating virtual contents relating to the exhibits, such as pictures, models, and animations, into the real environment, to increase sensory stimulation, improve display richness, and solve the problems such as inadequate explanation service. (2) The applications designing MAR guide with the hybrid tracking registration method and in combination with behavioral patterns of the users. (3) The applications introducing the heart flow mechanism into design of MAR system and proposing novel forms of museum education such as interactive narration and serious game, to create a deeper level of psychological immersion based on physiological immersion and realize value output of intangible assets, thus revealing deeper humanistic connotation from the dimension of user experience.

The article "A Survey of Museum Applied Research Based on Mobile Augmented Reality" was published in 2022. Journal: Comput Intell Neurosci.

### 3.1. MAR Applications Based on Sensory Stimulation

In museums, the important informal learning sites, the users may get information relying on interest tendency and independent behaviors; however, most people could not fully understand the additional information beside the showcase. Traditional visiting would reduce the value of exhibition. The core value of a museum is to provide high-quality information services; the cultural connotation could not only be presented to users by exhibition but also be attached with clear statements, attractive animations, and figurative 3D models, so as to display more details of the exhibits and integrate guide information and exhibits into the users' field of vision, thus meeting more information cognitive needs.

In some museums, certain valuable exhibits may have been damaged, and some ancient exhibits may be vulnerable and unsuitable for display; therefore, the visitors cannot fully view the cultural relics. 3D modelling in the AR system can completely restore the damaged cultural relics [31], showing the original freshness and vividness and enhancing the visitors' visual perception of the reality. Wang et al. [32] “reconstructed” ancient buildings in The Old Summer Palace such as the Water Observation and the Hall of National Peace with AR technology (Figure 7). For preventing murals from damage, Kenerdine reproduced the murals of Mogao Caves by AR. The Detroit Museum in the United States has become the first museum in the world to introduce Google's Project Tango AR technology, and the MAR application in the Detroit Museum showed the fish models after bone restoration (Figure 8). Barrile et al. [33] prepared 3D models of clay masks in the Regional Museum of Lipari, and the users can zoom in and view their details (Figure 9). Woniak and Poap [34] created a novel soft tree decision structure to make intelligent decisions about how to classify and evaluate the value of hard-to-identify cultural relic remains.

In order to improve the users' interaction and participation, Shaanxi History Museum designed cards of MAR cultural relics (Figure 10), and the users can view 3D cultural relics on the cards and listen to the audio commentary.

In addition to cultural relic restoration and cultural creation display by means of 3D reconstruction, AR can enhance sensory stimulation of the users and stimulate their curiosity for attention. Greci [35] used interactive graphics to highlight key details of figures, gestures, and objects and explain graphical implications (Figure 11). “Terra Fish” MAR displayed jellyfish species that do not exist in the sea of South Florida, to highlight the destructive effect of invasive species. Invitto et al. [36] took 3D images as visual stimuli in Museum of Educational Naturalism (Figure 12) and also took the calls of Tyrannosaurus and water sounds as auditory stimuli; the results proved that sensory stimulation and immersive experience can enhance the users' cognition, stimulate learning motivation, and also improve their neuroplasticity, recognition memory, and emotional engagement to varying degrees.

The article "A Survey of Museum Applied Research Based on Mobile Augmented Reality" was published in 2022. Journal: Comput Intell Neurosci.

### 3.2. MAR Guide Based on Behavioral Pattern

The existing museum voice guide system could obtain the locations of visitors by the radio frequency technology; it could play the audio explanation of cultural relics, but the contents are still boring, and the one-way output mode would also produce a fault between the visitors and exhibits. An MAR guide based on user behavior can plan reasonable visiting routes in advance [37], the real-time interaction with users can improve their observation and concentration, and also deepen their ability of art appreciation and aesthetic understanding. Dunleavy et al. [38] and McCall et al. [39] found that the users generally had excessive pursuit of sensory stimulation of AR, but ignored the exploration of real exhibits; however, Chang et al. [40] found in the analysis of behavior patterns that the visitors did not pay much attention to novel technologies, and the AR-guided mode could deepen the connection between the users and artworks.

Hammady et al. [41] designed an AR guide system based on user behavior feedback with the communication model; the feedback was obtained by the following methods: obtaining users' comments and emotions through interviews; determining the degree of participation and interest based on the visiting data; and analyzing visiting demands through social media. Lee and Park [42] designed a MAR guidance system for selective viewing according to points of interest with inertial trackers, which could guide the user to move to the next point of interest through directional indication, relative distance, and visual prompt (Figure 13). Capuano et al. [43] expanded the knowledge model based on the exhibits, performed sensory stimulation with MAR, and tracked the users' preferences through emotion detection, thus meeting their personalized cultural travel needs (Figure 14). Torres-Ruiz et al. [44] designed the Mexico Itinerary Recommendation System (Figure 15) based on information mining, beacon sensing, semantic processing, and machine learning; this system could extract the data of user preferences and visiting behaviors and perform semantic processing of the multidimension data set of exhibits, to obtain the context vectors under semantic recommendation, thus providing visiting decisions for the users by the machine learning algorithm. The testing found that technical acceptability and software practicability of this system could reach 80%. Wang [45] designed an AR mobile navigation system (Figure 16) based on the indoor positioning function of iBeacon and proposed four content recommendation mechanisms: interest recommendation, popular recommendation, mixed recommendation, and the expert recommendation. The system can analyze explicit interests through the basic information filled in by tourists in the early stage, infer the implicit interests of tourists by locating the user's location and time information, and finally provide personalized navigation suggestions through contextual reasoning.

The article "A Survey of Museum Applied Research Based on Mobile Augmented Reality" was published in 2022. Journal: Comput Intell Neurosci.

Hammady et al. [46] introduced a new narrative form, the Ambient Information Visualisation Concept (AIVC), into the design of AR museum applications, and set up a 3D virtual narrator of the King Tutankhamun to tell stories, display images, videos, and other related virtual information. They built a virtual war scene to provide users with an immersive space virtual experience (Figure 17). In addition, Hammady et al. [47] also mentioned that the behavior and information of the virtual tour guide are preset according to fixing themes, and more anthropomorphic free interaction based on artificial intelligence technology is not currently supported (Figure 18).

### 3.3. MAR Experience Based on Heart Flow Mechanism

AR can reshape exhibits as the “creation technology” and also realize “cultural reconstruction” of a museum, so as to make the users fully get into the cultural structure of the museum. The concept of heart flow refers to the mental state that the users fully invest their personal energy into certain activities. At the same time, Chauhan et al. [48] also emphasized that the streaming experience in the entertainment game center has a significant impact on user behavioral intentions. Virtual reality can make use of the sensory channel to create an all-round physiological immersion for the users and make them enter the above-mentioned state. However, Augmented Reality is half virtual and half real. The addition of virtual objects is to emphasize the cognition of reality, and the sense of physical immersion would be weak. In order to replace the forced infusion-type sensory stimulation, some researchers have introduced interactive narration and serious game into the MAR system, which can naturally introduce intangible cultural assets into the narrative plots or game mechanisms, and the interesting and novel interactive experience could make the users gradually lose their self-awareness of human-computer interaction and voluntarily move into the heart flow experience.

The article "A Survey of Museum Applied Research Based on Mobile Augmented Reality" was published in 2022. Journal: Comput Intell Neurosci.

Liestøl [49] introduced Trivia Game into MAR application of the ancient Roman road, to test the users' understanding of knowledge. Hammady et al. [41] introduced shooting games into MAR application of the Egyptian Museum (Figure 19), to enhance the visitors' impression of the cultural background. Krzywinska et al. [50] developed a “Tunnel escape class” MAR application of Telegraph Museum based on adventure games (Figure 20); the users may wear HoloLens and learn telegraph codes, repair communication cables, and complete various tasks with gesture interaction from the perspective of a new telegraph operator in the real bulletproof tunnel, so as to create information cognition for the users, and achieve emotional engagement. This system could produce a strong sense of participation and presence, but the technical usability index of gesture interaction is not quite ideal. Paliokas et al. [51] used the ARCore development kit in Unity to design the e-Tracer AR Application for the Greek Silver Museum. The application supports tourists to scan the cultural relic signs to display the 3D models of the cultural relics. Especially after the tourists visit the exhibition, the AR quiz game allows tourists to return to find and scan a certain cultural relic, which can get points and symbolic rewards and let tourists have the opportunity to reobserve the cultural relics and pay attention to details. These designs will stimulate more motivation for tourists to visit the exhibition (Figure 21). Fazio and Turner [52] introduced an AR narrative adventure game in the architectural space of intangible cultural heritage and designed seven plot nodes to be triggered, allowing tourists to actively explore virtual characters in the journey to experience the dramatic local culture. This form can be used to solving the problem of architectural a common “empty room” problem at space sites (Figure 22). Besides, the innovative and typical MAR application functions, major advances, and shortcomings mentioned in the paper in different countries and museums are summarized in the form of a table (Table 3).

## 4. Design of Mobile Augmented Reality Application for Museums

Museums cover all stages of human development. They preserve a considerable number of cultural and historical, scientific and natural heritages and carry intangible assets such as scientific knowledge, humanistic thoughts, experience, and skills. As the media, a museum plays an important role in disseminating information to the public. In the digital information age, the users have more visiting appeals. MAR can rebuild museums as the interactive and experiential cultural and educational sites. An ideal MAR system should display virtual information and stimulate the users' senses from a multidimensional perspective, provide precise spatial positioning and scene navigation for the users, and make them interact with the scenes and exhibits, thus forming a closed interaction loop of “users, exhibits and scenes.” Later, the design thought of MAR application will be discussed from virtual content design, navigation model design, and interaction mode design.

The article "A Survey of Museum Applied Research Based on Mobile Augmented Reality" was published in 2022. Journal: Comput Intell Neurosci.

### 4.1. MAR Content Design

The basic function of MAR application is to superimpose virtual information on real exhibits by means of multimedia forms such as text, picture, audio, video, 3D models, and model animation. The developers generally explain key information of cultural relics with text and audio, but they should reasonably control the amount of text information, and the contents should be professional and interesting. Pictures, videos, 3D models, and model animations can intuitively express the abstract concept, carry all microscopic and macroscopic images from plankton to stars, and help to improve the richness and aesthetic value of exhibits. The design thought of MAR virtual contents are proposed as follows based on the studies on MAR application design and testing:

1. Highlight the details of cultural relics with virtual information: highlight the local details of paintings and calligraphy works by means of zooming, highlighting strokes, or interactive icons, to enhance the visual effect of cultural relics, and shorten the time for information searching.
2. Attach dynamic elements to static cultural relics: dynamic elements can grant static works with fresh vitality, reproduce the previous glory of cultural relics and prosperous architecture, and also increase interestingness to the users' appreciation behaviors; in addition, human eyes can rapidly capture dynamic information on static works, so the dynamic information can play a role of highlighting the details and guiding the users.
3. Restore damaged historical relics with 3D models: since people are more compatible with 3D objects in terms of physical and psychological perceptions, the stereoscopic images can enhance the users' visual perception, and they may not fill the gap in reality with imagination but can intuitively experience the scenes that cannot be seen in real environment and even interact with them.
4. Display intangible cultural assets with video or animation: in addition to tangible cultural relics and exhibits, there would be a large number of intangible cultural assets, such as historical stories, cultural customs, skills, and experience in museums. Considering the fact that concrete images cannot present their cultural connotations, the developers can make use of videos or animations to present them to the users, such as telling historical stories by “scene reproduction,” describing human customs by “character stories,” and teaching skills and experience by “process deduction.”
5. Reduce complex interaction design and improve the comfort of application: the developers should simplify the interaction behavior, appropriately add interaction buttons, and make the users use their fingers as little as possible; the contents on the interface should be brief, clear, and focused, and the interactive functions should be easy to understand and operate.

The article "A Survey of Museum Applied Research Based on Mobile Augmented Reality" was published in 2022. Journal: Comput Intell Neurosci.

### 4.2. MAR Guide Design

We have summarized the design thought of MAR guide based on the case study. The guide framework consists of knowledge model, scene model, navigation model, and user model, in which, the knowledge model refers to the network model combining the existing exhibits with digital resources of the relevant cultures from the Internet dimension. In addition to the supply of digital resources for exhibits in the museums, the developers also collect cultural information and multimedia resources related to exhibits from the Internet, to connect resources and construct knowledge networks according to semantic tags. The combination of ontology resources and other digital resources can improve the added value of visiting, extend the breadth and depth of exhibits, and enhance the professionalism and interest of virtual information.

The scene model contains information of each exhibit from the physical, semantic, and virtual dimensions. The physical dimension refers to the spatial location of the exhibit, which can be used to construct a physical scene of “exhibit-exhibition area-exhibition hall-museum”; the semantic dimension refers to cultural and semantic tags of the exhibit, including exhibit's information and cultural attributes, while the virtual dimension refers to AR virtual contents and interactive elements designed for the exhibit.

The navigation model refers to a model constructed based on the context. The developers analyze the similarity between exhibits from a multidimensional dimension based on semantic contents of exhibits, to determine the locations of exhibits in multidimensional space; they also use special columns to set the selective attention weight, adjust the multidimensional space structure, and build a generalized context model, thus planning the visiting routes for different column topics in combination with the scene model and forming the navigation model.

The user model is used to store individualized data about interest preference of the users, including the static prior model and dynamic behavior model. With the static prior model, the data of age, gender, and cultural interest can be obtained from the basic information of the users, while with the dynamic behavior model, the preference data can be obtained through autonomous selection and passive recognition; autonomous selection refers to the behavior that the user actively selects the digital contents or marks the points of interest during the experience and passive recognition refers to the process of tracking user behavior data (eye tracking, gesture recognition, duration, and interaction times) with sensors, to parse the user preference data. Through adjusting user interest characteristics with the adaptive algorithm based on dynamic behavior data, the MAR navigation system can match with the navigation model according to user preferences, and appropriately add virtual information, to enable the users to get better visiting experience.

The article "A Survey of Museum Applied Research Based on Mobile Augmented Reality" was published in 2022. Journal: Comput Intell Neurosci.

In summary, the developers may take the following steps in the process of designing MAR navigation system: firstly, the developers may determine the virtual information of ontology resources and expand a knowledge model network for each exhibit; secondly, they may determine the base path according to the point information and virtual content of scene models connecting ontology resources of museums; thirdly, they may establish a navigation model and refine the visiting routes of different columns; and finally, they may analyze the basic information of the users, select the initial visiting route, change the navigation strategy in a real-time manner based on the dynamic behavior data, and replan the optimal navigation path.

### 4.3. MAR Museum Interaction Design

Sylaiou et al. [31] studied the sense of presence and degree of enjoyment of the users when visiting virtual museums and found a close correlation between the high level of sensible presence and visiting satisfaction; namely, the users may have a positive experience when interacting with an AR system. Compared with virtual reality, an MAR system is relatively weak in the sense of immersion and presence, and after experimenting with the new technology, the users' initiative and sense of participation would gradually decrease. Therefore, the researchers have introduced novel interaction mechanisms, such as serious game and interactive narration, into MAR design, so as to make the users enjoy the visiting by participating in the experience, stimulating their curiosity and pleasure, and enhancing their intangible cultural awareness.

Serious game, as a form of game for educational training with the essential characteristics of traditional games, can be taken as a carrier for publicizing intangible assets of museums, including historical information and cultural thoughts. Traditional games are generally divided into adventure, simulation, action, casual, puzzle, and RPG games, which can be determined in accordance with the types of cultural relics, to develop MAR interaction modes with novel forms and unique contents. For example, based on RPG and interactive storytelling, the developers can design game plots referring to humanistic stories, to make the users experience the legendary life of historical figures from the first-person perspective, with stronger sense of involvement and engagement. Based on adventure games, the developers can set thrilling adventure tasks, such as famous battles in history; based on action games, the developers can integrate the techniques of fruit pit carving, paper cutting, and colored embroidery into interactive actions, making the users participate in the making of artworks through virtual interaction; and based on puzzle games, the developers can design quizzes to deepen the users' understanding and impression of the culture.

The article "A Survey of Museum Applied Research Based on Mobile Augmented Reality" was published in 2022. Journal: Comput Intell Neurosci.

## 5. Conclusion and Future Work

At present, the limited physical space in museums cannot meet the increasing cultural needs of the public; MAR can reconstruct a museum from the virtual dimension and the users' perspective, to get rid of inadequate explanation and single way of display, enhance the richness and aesthetic value of the exhibits, and design individualized visiting routes for all users, thus offering participatory and immersive visiting experience.

Domestic and foreign researchers and developers have started their studies on MAR application in museums. This article first briefly summarizes the development process of core MAR technologies and their application in museums; then classifies and summarizes the application cases of MAR from the perspective of application functions and briefly describes the design contents and application effect; finally, it provides certain ideas and suggestions for content design, user guide, and interactive experience of MAR system based on previous studies and combined with the dimensions of application usefulness, technology usability, experience enjoyment, and participation purpose.

Firstly, a museum MAR system can adopt the hybrid tracking registration method based on the vision and hardware; the rapid positioning of sensors can reduce system delay; and the optimization of image recognition algorithm can greatly improve the registration precision and system robustness. From the perspective of real-time interaction, handheld mobile devices can be used for 6DOF interaction by means of touch control, while head-mounted devices should perform interaction by gestures; therefore, the users shall first learn certain gestures. In addition, due to the occlusion of gestures, gesture recognition precision should be improved in combination of a lot of depth data. Furthermore, by virtue of the closeness to eyes and a strong sense of immersion, head-mounted devices are the application devices most in line with the MAR concept; however, due to the high price of head-mounted devices and the high cost of learning, handheld mobile devices have more potential at present, and most of the MAR systems are designed based on handheld mobile devices.

The article "A Survey of Museum Applied Research Based on Mobile Augmented Reality" was published in 2022. Journal: Comput Intell Neurosci.

In terms of functional design, the previous application cases and evaluation research showed that with the software development kits provided by engine companies such as Unity3D and Wikitude, the developers can easily design virtual contents and complete virtual-real fusion. MAR that can superimpose virtual objects on real exhibits to enhance the users' sensory stimulation has been widely used, but the research on individualized MAR navigation and innovative MAR interaction is still in progress. In the future, the researchers may intensively study the individualized navigation model based on user interest preference, or intelligent audio navigation system established based on user behaviors. Developers may also integrate the game design concept into system development, and innovatively combine gameplay with the features of cultural relics, to design novel MAR interaction or explore more immersive interaction modes from psychological dimensions of the users.

## Figures and Tables

**Figure 1:** System architecture of Mobile Augmented Reality.

**Figure 2:** Classification of Augmented Reality tracking registration technology.

**Figure 3:** “Talking Celts” markers (a) and recognition effects (b) [10].

**Figure 4:** (a, b) The marking method based on markers; (c, d) the marking method based on natural features [20].

**Figure 5:** Navigation interface (a) and beacon guide for each floor (b) [23].

**Figure 6:** Freeze view menu bar (a) and auxiliary axis button (b) [27].

**Figure 7:** Water observation site of The Old Summer Palace (a) and Augmented Reality effect (b) [32].

**Figure 8:** Users can scan the fish bones to see the complete fish (image source: https://vr.poppur.com/AR/3462.html).

**Figure 9:** Mask reconstruction based on digital technology [33].

**Figure 10:** Card of terra-cotta figures of Tang dynasty in Shaanxi History Museum (this picture comes from the Internet).

**Figure 11:** Watch and listen section (a) and active areas section (b) [35].

**Figure 12:** 3D stereoscopic image of plankton (a) and Tyrannosaurus (b) [36].

The article "A Survey of Museum Applied Research Based on Mobile Augmented Reality" was published in 2022. Journal: Comput Intell Neurosci.

**Figure 13:** Navigation map (a) and Additional instructional information (b) [42].

**Figure 14:** Associated knowledge graph of the “The Procession to Calvary” [43].

**Figure 15:** Exhibition identification (a) and tour guide screen (b) of Mexico itinerary recommendation system [44].

**Figure 16:** Newly visited tour route and the new recommended tour routes of hybrid recommendation [45].

**Figure 17:** Scene of “The Battle” (a) and the participant (b) [46].

**Figure 18:** MuseumEye—the MR virtual guide system and levels of interaction [47].

**Figure 19:** “Horus” game interface [41].

**Figure 20:** “Tunnel escape class” MAR application of telegraph museum [50].

**Figure 21:** Typical quiz question (a) and AR question which makes tourists to find (b) [51].

**Figure 22:** The pictures of the heritage engagement project “Skullduggery” [52].

**Table 1:** Natural feature-based tracking registration method and its realization principle [11].

Natural feature-based tracking registration method	Realization principle
Edge detection	Project 3D model onto a 2D image, matching with the features of the corresponding edge, and calculate 3D camera motion between frames based on 2D displacement of the corresponding feature, to realize pose tracking [12]

Point of interest tracking	Identify the features of target points from the image database, and then save the location and virtual information; extract feature points in the current view, and match them with the features in the database, to estimate the camera pose [13]

Template matching	Through recognizing the texture information in the camera view, match with the most relevant images in the image database, to estimate the camera pose [14]

Optical flow tracking	Under the premise of the constant spatial projection intensity, the physical point in video sequence can be tracked through measuring the speed of pixel position change in the path of projecting a 3D object onto a 2D plane, so as to complete pose tracking [15]

Depth imaging	Generate depth images with the reference pixel value of the distance between the camera view and the object, and integrate the depth images with RGB images for estimating the camera pose [16]

Model-free tracking	This method can realize tracking without a model or database; the reconstruct 3D structure of the images through tracking the focal length, the rotation matrix, and the translation vector of the camera, and perform triangulation between the corresponding points of each image, to calculate the camera pose [17]

**Table 2:** Support rate of MAR development tool, 2019 AWE AR expo and main functions realized by SDK.

MAR development tool	Support rate (%)	Main functions
ARKit	73	2D image recognition and tracking, 3D object recognition and tracking, environmental probe, character occlusion, motion capture, face detection and tracking, multiperson sharing, etc.
ARCore	68	Image recognition and tracking, motion tracking, light estimation, environment understanding, cloud anchor, etc.
Unity's AR foundation	64	It is the re-encapsulation of ARKit, ARCore and SenseAR, and supports the functions in the framework of ARKit, ARCore, and SenseAR
Vuforia	40	Image recognition and tracking, object recognition and tracking, VuMarks mark recognition and tracking, environment tracking, cylinder recognition, plane recognition, equipment tracking, cloud recognition, etc.
AR framework of unreal	27	Support the core functions in ARKit and ARCore framework
Facebook spark AR	23	Image recognition, face detection and tracking, multilevel recognition, multitarget tracking, compatibility with messenger communication applications, etc.
Amazon Sumerian	20	Support the core functions in ARKit and ARCore framework
Snap lens studio	17	Body tracking, multiobject detection, 3D body mesh, cloth simulation, social sharing, gesture recognition, voice machine learning, etc.
Adobe project aero	17	Display 2D/3D interactive art works in the real world
Wikitude	14	Micro AR Clouds, real-time tracking (unmarked SLAM function), image recognition and tracking, object recognition, AR function based on fixed location, etc.
EasyAR	12	Motion tracking (SLAM), 3D object tracking, screen recording, AR Cloud, image recognition and tracking, gesture recognition, etc.

The article "A Survey of Museum Applied Research Based on Mobile Augmented Reality" was published in 2022. Journal: Comput Intell Neurosci.

**Table 3:** Research on the application of augmented reality in museums.

Research object	Museum/country	Main function	Main advances	Application disadvantages (if mentioned in the article)	Researchers
Augmented Reality system of The Old Summer Palace	The Old Summer Palace/ China	The software uses augmented reality technology to digitally reconstruct the ruins of The Old Summer Palace, and uses visual effects to more vividly and intuitively restore the prosperous scene previously.	Three forms of fixed-point observation, handheld PDA, and wearable HMD are adopted to bring different outdoor display effects to users:	The display mode of the handheld PDA is limited by the display screen, image resolution of which is low, and the stereoscopic effect cannot be presented. In addition, the computing resources in this form are limited, and the system performance will be reduced in terms of image compression, transmission, and registration accuracy.	Wang et al. (2006) [32]
			a) When using the fixed-point observation form, the user can adjust the angle of view zoom, lens zoom, light intensity, and can play video and sound		
			b) Tourists can use the PDA Augmented Reality system to view digitally reconstructed attractions from a distance and have a high degree of freedom.		

Augmented Reality (AR) guide for religious museum	Museo Diocesano of Milan/ Italy	a) Explain the artwork and point out the relevant collections	The software contains explanation videos of relevant artworks, and the key parts are marked with virtual icons to help tourists understand the deep meaning of religious paintings in a more convenient and intuitive form.		Greci (2016) [35]
		b) Provide visitors with 3D models of exhibits			
		c) Provide online communication area for tourists			

The app of Augmented Reality in education naturalistic museum (MAUS)	Museum of Environment, University of Salento/ Italy	The project presents visitors with 2D/3D images and sounds of natural creatures, bringing visual and auditory perceptual stimulation to them.	This research uses Augmented Reality and Virtual Reality technology to create 2D and 3D virtual images for natural creatures in museums and stimulates users' learning interest and learning ability by creating multisensory stimulation.		Invitto et al. (2014) [36]
The “Horus” AR game	Egyptian museum in Cairo/ Egypt	Let tourists understand the historical and cultural background of ancient Egypt through shooting games.	The study analyzes feedback factors in the communication model of the museum's AR software and introduces visitors to the history and culture of ancient Egypt in the form of an AR game.		Hammady et al. (2016) [41]
Augmented Reality-based guidance system	Art Museum/ Korea	The application provides visitors with guided paths for selective viewing and provides multimedia information on relevant exhibits.	a) Guide visitors to exhibits of interest by displaying relative directions, distances, and visual cues on the screen		Lee et al. (2007) [42]
			b) Provide visitors with additional multimedia information about exhibits		

Fruizione innovativa dei beni artistici e culturali (FIBAC)	Museum exposition related to Flemish paintings/ Italy	The project extends the knowledge network model of the exhibits to present multimedia resources to visitors in the form of Augmented Reality	This research combines augmented reality and semantic technology, constructs knowledge model network through cultural artefact modelling, knowledge deduction modelling, and multimedia modelling, and extends other cultural resources from the two dimensions of similarity and difference.		Capuano et al. (2016) [43]
Itinerary recommendation system	Museums in Mexico/ Mexico	The project provides tourists with the best indoor and outdoor tour routes by analyzing data such as user preferences, expert recommendations, public opinion, and tour experience.	The system uses information mining, beacon sensing, semantic processing, machine learning, and other technologies to design a hybrid method to provide users with intelligent tour decisions and improve user experience through multidimensional analysis.	Some behaviors of the users are not taken into account in this project, such as not all routes offer children's transport and some places do not offer activities for singles.	Torres-Ruiz et al. (2017) [44]
AR mobile navigation system	The Mackay Memorial Museum/ China Taiwan	The AR mobile navigation system identifies the pictures of the exhibits according to the unmarked method and uses iBeacon indoor positioning to track the location of tourists. Visitors can choose four content recommendation mechanisms: interest recommendation, popular recommendation, mixed recommendation, and the expert recommendation for navigation, and can scan the pictures of the exhibits to browse related 3D virtual content and navigation information for exhibits.	a) This study proposes a positioning mechanism that adjusts the sensing value of iBeacon according to distance, which supports more stable and accurate indoor positioning function.		Wang (2018) [45]
			b) This study proposes content recommendation services under four navigation recommendation mechanisms: interest recommendation, the hotspot recommendation, hybrid recommendation, and the expert recommendation. Among them, the hybrid recommendation method combines the explicit interests inferred from the information of user and the latent interests predicted by users' browsing behavior, and offer personalized navigation suggestions in real time according to the context.		

MuseumEye MR application	Egyptian Museum/ Egypt	a) The virtual guide can speak to the visitor and provide various types of visual information such as videos, images, 3D visualisations of artefacts and spatial sound effects.	While most studies in this field use the AR guide system only as a tool to support the guided experience of museums, this study redesigned the functions of AR guide system by analyzing the background of museum experience, the function of guide role, and the different needs of users, and through multidimensional interactions, guided storytelling, and gameplay mechanics adds to the fun. At the same time, the system enhances the experience of traditional museums by replacing human tour guides with virtual models and emphasizes multilayer interaction, multimedia display, user interface design, and practicality in the museum scenarios to enhance the guidance of tourists.	a) Equipment level: glasses have narrow field of view, and glasses are too heavy	Hammady et al. (2021) [47]
		b) The game named “KnowledgeScale game” encourages visitors to discover hidden secrets and clues in the virtual relics.		b) Content level: more content needs to be displayed and the exhibit menu is needed set in the system. Furthermore, the model is slightly different from the real exhibit.	
				c) Interaction level: the direction of the behavior is not clear, and the system needs more guidance UI or auxiliary instructions.	

“Tunnel escape class” MAR application	Porthcurno Telegraph Museum/ England	Users wear HoloLens glasses in a real bulletproof tunnel, learn telegram passwords, repair communication cables from the perspective of telegraph recruits, and use gesture interaction to complete various tasks.	This research integrates the constructivist model of education into the museum field, introduces the elements of “escape room” games into the MAR application, and creates a mission-based and narrative-based museum education and entertainment tour experience for tourists.		Krzywinska et al. (2020) [50]
e-Tracer AR application	Silversmithing Museum/ Greece	a) Users scan images of cultural relics to get an introduction to the exhibits and can preview the 3D model of the cultural relics and zoom in and out of the cultural relics to study the details.	a) Compared with the audio guide system, the AR system is more suitable for tour experience and has a stronger sense of immersion and interaction.	a) Interaction level: the visual metaphor of the time bar is not clear.	Paliokas et al. (2020) [51]
		b) The quiz game is divided into “detection game” and “AR search game,” the latter of which will allow visitors to return to find and scan an item for points and token rewards.	b) Small cultural relics are inconvenient for tourists to view in all directions and at close range in the cabinet. This application uses the unmarked identification method instead of QRC identification and provides a 3D model that can be enlarged and solve the above problem.	b) Functional level: in the case of insufficient light, the system has errors in the positioning of the user's position and direction.	
			c) The AR Q&A system integrates AR experience, scavenger hunt game mechanics and self - assessment of new knowledge, allowing tourists to reobserve cultural relics and pay attention to details. AR games will stimulate more motivation for tourists to visit the exhibition		

The heritage engagement project “Skullduggery”	Old Government House (intangible cultural heritage)/ Australia	“Games for Cultural heritage experience,” an AR application based on an adventure narrative game, takes the old government house intangible cultural heritage (ICH) as the game environment, and sets seven plot nodes to trigger in combination with the user journey. Visitors are provided with a cultural heritage-based narrative experiential game that addresses the “empty room” problem encountered in heritage sites such as historic buildings.	This study uses the real scene of the site as the spatial background of the adventure game and proposes a new AR display method for Intangible Cultural Heritage (ICH), which can well display “the spirit of a place” and solve the problem of “empty rooms,” which enhances the visitor's sense of history and presence.	Interaction level: limited triggers and mediocre navigation	Fazio et al. (2020) [52]

The article "A Survey of Museum Applied Research Based on Mobile Augmented Reality" was published in 2022. Journal: Comput Intell Neurosci.

## Data Availability

The data used to support the findings of this study are available from the corresponding author upon request.
